This article has been retracted.

# A case of meningitis due to *Achromobacter xylosoxidans* in a child with a polymalformative syndrome: a case report

**DOI:** 10.11604/pamj.2021.39.124.29794

**Published:** 2021-06-15

**Authors:** Mehdi Borni, Mohammed Znazen, Fatma Chaker Borni, Mohamed Zaher Boudawara

**Affiliations:** 1 Department of Neurosurgery, University Hospital Center Habib Bourguiba, Sfax, Tunisia,; 2 Department of Obstetrics and Gynecology, University Hospital Center Hedi Chaker, Sfax, Tunisia

**Keywords:** *Achromobacter xylosoxidans*, meningitis, antibiotics, case report

## Abstract

Achromobacter xylosoxidans (AX), also called alcaligenes xylosoxidans, is an aerobic, non-fermenting mobile, gram-negative bacillus which was first isolated in an otorrhea samples in 1971. Infections with these species are quite rare and have often been described in immunocompromised and in premature infants. However, very few cases of meningitis related to AX have been reported in the literature. The authors report a new case of meningitis due to AX in a 45-day-old female infant with polymarformative syndrome meningitis was confirmed by a cyto-biochemical analysis and culture of the cerebrospinal fluid and was treated by antibiotherapy. Hydrocephalus was managed initially with external ventricular drainage followed by a ventriculoperitoneal shunt after rigorous cerebrospinal fluid (CSF) sterilization, with good clinical and radiological outcomes. The prompt and adequate antibiotic adjustment following bacterial isolation has been shown to rapidly modify the clinical outcomes.

## Introduction

*Achromobacter xylosoxidans* (AX), also called alcaligenes xylosoxidans, is an aerobic, non-fermenting mobile, gram-negative bacillus [1] which was first isolated in an otorrhea sample and described in 1971 [1]. The mode of patients´ contamination is still unknown. Infections with these species are quite rare and have often been described in immunocompromised and in premature infants with low birth weight or young children [2,3]. However, very few cases of meningitis related to AX have been reported in the literature previously usually in patients with accompanying sepsis after neurosurgical procedures or penetrating head traumas [4].

Here the authors report a new case of meningitis due to AX in a 45-days-old female infant with polymarformative syndrome. Meningitis was confirmed by cyto-biochemical analysis and culture of the cerebrospinal fluid and was treated by antibiotherapy. Hydrocephalus was managed initially with external then internal shunt, with good clinical and radiological course. The authors proceed with an over review of the literature regarding this rare entity and its recent management.

## Patient and observation

**Patient information:** a 45-day-old female infant (birth weight 2800 grams) was admitted to our Neurosurgical Department for macrocrania associated to intermittent fever. She was born by caesarean section at 37 weeks, after normally developed and followed pregnancy out of consanguineous marriage. The mother's age at the pregnancy was 38 years old with history of 3 previous pregnancies and 2 healthy stillborns. Ventriculomegaly associated to a lumbosacral spina bifida were diagnosed on foetal morphology ultrasound. At birth, the general condition of the baby was satisfactory. However, the mother noticed a progressive increasing head circumference. At the age of 40 days of life, the baby presented a fever with rapid onset without any episode of vomiting or epileptic seizures.

**Clinical findings:** at presentation, the baby was not well reactive and her head circumference diameter was 42 cm (2 standard deviations or more from the normal for female infant) contrasting a circumference of 36 cm at the age of 22 days. Neurological examination revealed cranial suture disjunction, blatant axial hypotonia with clenched fists and flexed elbows and bulging anterior fontanellle. The rest of physical and neurological examination showed also a flaccid paraplegia and lumbosacral spina bifida aperta (myelomeningocele), measuring 10 cm in diameter associated to a tuft of hair below the pouch. No CSF leak or breach from the myelomeningocele was noticed. The cardiorespiratory check-up was satisfactory. Chest X-ray had normal appearances.

**Diagnostic assessment:** routine biological screening showed an increase in C-reactive protein at 102 mg / L (normal <3.2), fibrinogen at 6.5 g/L (normal 2-4), and neutrophils at 17000 cells/mm^3^ (normal 1800-7500). Transfontanellar ultrasound using 7.5 MHz transducer showed moderate ventriculomegaly (lateral ventricular diameter between 12-15mm) (Figure 1). A Full Body magnetic resonance imaging scan (MRI) revealed a type I Chiari malformation associated to triventricular hydrocephalus with no signs of transependymal edema. Spinal cord imaging showed an extensive cervico-dorsal syrinx from C7 to D5 and lumbosacral myelomeningocele with low-lying spinal cord (Figure 2).

**Figure 1:** mid-anterior ultrasound scans showing a moderate ventriculomegaly (yellow arrows) with abnormally large lateral ventricles (especially ventricular atrium and occipital horns; lateral ventricular diameter between 12-15 mm) and the third ventricle; the scans were performed using 7.5 MHz transducer through anterior fontanelle approach; note the absence of low-level internal echoes that are consistent with debris/pus within the ventricles

**Figure 2:** full body magnetic resonance imaging scan at presentation: (A, B) axial T1-weighted image and coronal T2-weighted image showing hydrocephalus; C) sagittal T2-weighted image showing downward displacement of the cerebellar tonsils beneath the foramen magnum into the cervical spinal canal (type I chiari malformation; yellow arrow) as well as a cervico-dorsal syrinx (white arrow) C7 to D5; D) sagittal full body scan showing lumbosacral myelomeningocele (red arrow)

**Therapeutic intervention:** faced with the presence of spina bifida, lumbar puncture was not feasible. A transfontanellar ventricular puncture was performed. It has revealed a turbid cerebrospinal fluid. Cyto-biochemical analysis revealed an increase in white cells at 88, deep hypoglycorrhachia (0.005 mmol/L) and high CSF protein concentration at 2.13 g/L. Incubation in an atmosphere of 10% carbon dioxide ravealed positivity of the CSF culture on blood agar and chocolate agar plates. The concerned bacterium was identified using classic Gram stain showing a Gram-negative bacillus, oxidase + and catalase + concluding to a multi-resistant agent: *Achromobacter Xylosoxidans* (AX) (Figure 3). The infant had an external ventricular drainage (EVD) and put under empiric antibiotic therapy based on Cefotaxime (200mg/Kg/day in 4 divided doses) associated to Vancomycin (80 mg/day). Later, antibiogram study (Table 1) revealed an impressive antibiotic resistance pattern. An accidental removal of the EVD took place 9 days later, requiring a new set-up of the shunt. A second CSF cyto-biochemical analysis showed a persistence of hypoglycorrachia, high CSF protein concentration, and the same strain (AX) on the bacterial culture. Thus, antibiotic therapy was switched into a combination of Imipenem (400mg/day in 4 divided doses) with Vancomycin (60 mg/Kg) after checking the new antibiogram (Table 2). Cefotaxime was withdrawn after 7 days (because of antibiotics resistance pattern). The infant´s neurological condition was stable but CSF was still turbid and persistent abnormalities in CSF formula as well as the same germ were noticed. External ventricular drainage (EVD) was changed in the contralateral frontal ventricular horn after 30 days of parenteral antibiotic therapy based on Imipenem and Vancomycin. Cerebrospinal fluid (CSF) microbiological examination was repeated twice, showing no germ.

**Figure 3:** A) growth of *Achromobacter xylosoxidans* seen after 24 hours of incubation at 37°C on blood agar and chocolate agar plates, the colonies are smooth, glistening, low convex and non-lactose fermenting; B) classic gram stain image showing gram-negative *Achromobacter xylosoxidans* (blue arrow) with neutrophils (black arrow)

**Table 1:** first antibiotic susceptibility pattern of *Achromobacter xylosoxidans* isolated from cerebrospinal fluid culture

UHC Habib Bourguiba of Sfax-Clinical Microbiology Laboratory					
Antibiogram					
Requesting department: neurosurgery					
Sample: cerebrospinal fluid					
Culture: *Achromobacter xylosoxidans*					
Antibiotic	Interpreted result	MIC	Diam	Diam range	MIC range
Ampicillin 10μg	Resistant	128	6	16 - 21	2 - 8
Amoxicillin-clavulanite acid 20-10μg	Resistant			16 - 23	2 - 8
Ticaracillin-clavulanite acid 75-10μg	Sensitive	<0.0313	40	22 - 24	8 - 16
Piperacillin 30μg	No critical values			0 - 0	0 - 0
Piperacillin-tazobactam 30-6μg	No critical values			0 - 0	0 - 0
Cefalexin 30μg	Resistant	128	6	12 - 18	8 - 32
Cefoxitin 30μg	Resistant			15 - 22	8 - 32
Cefuroxime IV 30μg	Resistant	>256	6	22 - 25	4 - 8
Cefexim 5μg	No critical values			0 - 0	1 - 2
Cefotaxime 30μg	Resistant			0 - 0	1 - 2
Ceftazidime 30μg	No critical values			0 - 0	4 - 8
Cefepime 30μg	Resistant	>32	14	19 - 21	4 - 8
Aztreonam 30μg	Resistant	>512	6	21 - 23	4 - 8
Ertapenem 10μg	Resistant			26 - 28	0.5 - 1
Imipenem 10μg	Sensitive	<2	26	17 - 24	2 - 8
Meropinem 10μg	Sensitive	<0.125	37	15 - 22	2 - 8
Gentamicin 10μg	Resistant	128	6	16 - 18	2 - 4
Tobramycin 10μg	Resistant	128	6	16 - 18	2 - 4
Amikacin 30μg	Resistant	>256	6	15 - 17	8 - 16
Netilimicin 10μg	Resistant	>256	6	19 - 21	2 - 4
Norfloxacin 10μg	No critical values			0 - 0	0 - 0
Ciprofloxacin 5μg	No critical values			0 - 0	0.25 - 0.5
Trimethoprim 5μg	Resistant			12 - 16	4 - 8
Fosfomycin 200μg	No critical values			0 - 0	32 - 32

MIC: minimum inhibitory concentration; Diam: diameter

**Table 2:** second antibiotic susceptibility pattern of *Achromobacter xylosoxidans* isolated from cerebrospinal fluid culture (9 days later and after the new set-up of the external ventricular drainage)

UHC Habib Bourguiba of Sfax-Clinical Microbiology Laboratory					
Antibiogram					
Requesting department: neurosurgery					
Sample: cerebrospinal fluid					
Culture: *Achromobacter xylosoxidans*					
Antibiotic	Interpreted result	MIC	Diam	Diam range	MIC range
Ampicillin 10μg	Resistant	>64	8	16 - 21	2 - 8
Amoxicillin-Clavulanite acid 20-10μg	Intermediate	>2	22	16 - 23	2 - 8
Ticaracillin 75μg	Sensitive	0.25	34	22 - 24	8 - 16
Ticaracillin-Clavulanite acid 75-10μg	Sensitive	0.25	34	22 - 24	8 - 16
Piperacillin-Tazobactam 30-6μg	No critical values			0 - 0	0 - 0
Mecillinam 10μg	Resistant	512	6	18 - 22	2 - 8
Cefalexin 30μg	Resistant	128	6	12 - 18	8 - 32
Cefuroxime IV 30μg	Resistant	>256	6	22 - 25	4 - 8
Cefexim 5μg	No critical values			0 - 0	1 - 2
Cefotaxime 30μg	Resistant			0 - 0	1 - 2
Ceftazidime 30μg	No critical values			0 - 0	4 - 8
Aztreonam 30μg	Resistant		6	21 - 23	4 - 8
Ertapenem 10μg	Sensitive	<0,125	32	26 - 28	0.5 - 1
Imipenem 10μg	Sensitive	<2	26	17 - 24	2 - 8
Meropinem 10μg	Sensitive	<0,125	37	15 - 22	2 - 8
Gentamicin 10μg	Resistant	64	8	16 - 18	2 - 4
Tobramycin 10μg	Resistant	32	10	16 - 18	2 - 4
Amikacin 30μg	Resistant	128	9	15 - 17	8 - 16
Netilimicin 10μg	Resistant	256	7	19 - 21	2 - 4
Nalidoxic Acid 30μg	Resistant	>16	14	15 - 20	8 - 16
Norfloxacin 10μg	No critical values			0 - 0	0 - 0
Ciprofloxacin 5μg	No critical values			0 - 0	0.25 - 0.5
Trimethoprim + Sulfamides	Sensitive	<0.0313	34	10 - 16	2 - 8
Colistin 50μg	Resistant	3		0 - 0	2 - 2

MIC: minimum inhibitory concentration; Diam: diameter

**Follow-up and outcomes:** follow-up computed tomography (CT) scans were performed weekly to assess hydrocephalus and the catheter´s placement (Figure 4). The latest CT scan showed a decreased ventricular dilatation (Figure 4D). Our baby received a total of 34 days of antibiotic therapy combining Imipineme and Vancomycin, followed by oral relay using Trematoprim/Sulfamethoxazole (TMP/SMX) combined to intravenous Imipenem for two weeks. A ventriculoperitoneal shunt in the left ventricular atrium was then performed in view of the normality of CSF formula and its sterility. The CSF examination collected during surgery and 8 days postoperatively was normal. The infant received only TMP/SMX orally after surgery for two weeks with good clinical outcome. The baby was followed-up with a favorable course. She was discharged from our department in apyrexia after stabilization of her head circumference and disappearance of both axial hypotonia and bulging anterior fontanelle.

**Figure 4:** head CT scan slides at different time points following ventricular drainage: A) axial CT slide (brain window) showing hydrocephalus; (B,C,D) axial CT scan slides (brain window) 2 weeks (with biparietal subdural hygroma; yellow arrows), 3 weeks (without biparietal subdural hygroma) and 5 weeks (relocation of subdural hygroma; yellow arrows) after right external ventricular drainage (blue arrow); E) axial CT scan slide (brain window) showing the new left external ventricular drainage; F) axial CT scan slide (brain window) 2 days after ventriculoperitoneal shunt in the left atrium (red arrow) and before the discharge of the infant

**Patient perspective:** during hospitalization and at the discharge, the patient´s parent was delighted with the care.

**Informed consent:** the patient´s parent was informed about the report, why her case was peculiar and the authors’ interest in publishing her case. She gave informed consent to allow the authors to use her case for this case report.

**Patient's consent:** informed consent was obtained from the patient´s parent for us to use the case.

## Discussion

*Achromobacter xylosoxidans* (AX), also called alcaligenes xylosoxidans, is an aerobic, non-fermenting mobile, gram-negative bacillus [1]. Various species have been isolated from water sources and human gastrointestinal tract. However, it is not clear whether it represents physiological components of endogenous human flora. Infections with AX are quite rare and have often been described in immunocompromised patients and in premature infants or young children [2,3]. Excluding cystic fibrosis, infections reported include septicemia [3,4], urinary tract infections [5], osteomyelitis [6], conjunctivitis [7] or endocarditis [8]. However, very few cases of meningitis related to AX have been reported previously [9]. Two teams [10,11], in the 1970s, presented observations without taxonomic certainty. Nanmyak *et al*. [12] in 1985 reported infection in a 33-week premature baby with respiratory distress and hyperthermia complicated by meningeal involvement. This case was treated with carbenicillin at a dose of 1 g every 6 hours; however, the child developed hydrocephalus and died on day 47. Other report of six cases of cerebral ventriculitis, probably acquired in hospital, was reported in 1978 [13]. To our knowledge, our case seems to be the first to associate meningitis related to AX with polymalformative syndrome and good outcomes.

Genotypic studies show that each patient may be colonized with different strain. Cross-transmission is rare apart from transmission within siblings [14]. However, some studies showed that patients can be colonized by the same genotype´ strains, thus suggesting possibility of direct cross-transmission [15]. In our case, contamination mode was not well established as our patient did not express any respiratory, cardiac or even digestive signs of infections as well as her myelomeningocele which was dry and well covered at admission. The search for immune deficiency in our patient has been negative.

*Achromobacter xylosoxidans* (AX) is naturally resistant to many antibiotics: cephalosporins (except ceftazidim), aztreonam and aminoglycosides [3,16]. In our case there were no critical values to assess resistance to ceftazidim but the minimum inhibitory concentration (MIC) for gentamicin was 128 and exceeded 512 for aztreonam. Furthermore, acquired resistance is frequent [14,17,18]. Resistance of AX to antibiotics raises many questions among bacteriologists and clinicians. This resistance may be the result of enzymatic inactivation mechanisms of antibiotics, modification or protection of the antibiotic’s target, impermeability, or active efflux. Resistance phenotypes of clinical strains as well as our current knowledge concerning antibiotic resistance of non-fermenting gram-negative bacillus have led to search for efflux systems in this species. Acquired resistance is very common in clinical strains.

Several antibiotic sensitivity studies indicate that piperacillin with tazobactam and carbapenems are most frequently active on AX [16,18]. In our case there were no critical values to assess sensitivity to piperacillin and tazobactam and AX was sensitive to imipenem and meropenem (MIC <2 and <0.125, respectively). Recent studies and reports showed that AX could harbor various mobile genetic elements carrying genes for antibiotic resistance: plasmids, insertion sequences, integrons and transposons [19].

Faced with the escape of AX to advances in therapy by the adaptation mechanism, other scientists sought to eliminate this bacterium. Ma *et al*. reported the discovery of potential treatment [20]. A medical approach that is continually being developed to fight microbes uses phage therapy. This includes the involvement of lytic bacteriophages, which are specific to bacteria so that it can only target and eliminate these cells. In their report, these authors admit that many phages were discovered previously and totally sequenced, including phiAxp-1 and JWDelta. In their trail, a new specific phage was discovered called phiAxp-3. It may use any exposed lipopolysaccharides on bacterium as a receptor to try to bind to and enter the cell [20].

All these features demonstrate that therapeutic management of these agents may be difficult because AX is often very resistant to many antibiotics; a large number of isolates are still susceptible to cotrimoxazole, carbapenems and antipseudomonal penicillins, which are considered to be the treatment modalities of choice [3]. This is concordant somehow with our case in which our infant received a total of 34 days of antibiotic therapy combining imipineme and vancomycin, followed by oral relay using TMP/SMX combined to intravenous Imipenem for two weeks.

## Conclusion

Searching for unusual or atypical microorganisms when meningitis occurs in patients with such severe comorbidities cited above or in case of polymalformative syndrome in young infant with preterm birth is with extreme importance. The prompt and adequate antibiotic adjustment following bacterial isolation has been shown to rapidly modify the clinical outcomes.
